The article "Identification of hub genes and construction of prognostic nomogram for patients with Wilms tumors" was retracted in 2023. Reasons: errors in the cell lines or tissues; unreliable results or conclusions; concerns about the data.

# Identification of hub genes and construction of prognostic nomogram for patients with Wilms tumors

**DOI:** 10.3389/fonc.2022.982110

**Published:** 2022-10-21

**Authors:** Lei Lou, Luping Chen, Yaohao Wu, Gang Zhang, Ronglin Qiu, Jianhang Su, Zhuangjie Zhao, Zijie Lu, Minyi Liao, Xiaogeng Deng

**Affiliations:** ^1^ Department of Pediatric Surgery, Sun Yat-Sen Memorial Hospital, Sun Yat-Sen University, Guangzhou, China; ^2^ Department of Pediatric Surgery, The Third Affiliated Hospital of Guangzhou Medical University, Guangzhou Medical University, Guangzhou, China; ^3^ Guangdong Provincial Key Laboratory of Malignant Tumor Epigenetics and Gene Regulation, Sun Yat-Sen Memorial Hospital, Sun Yat-Sen University, Guangzhou, China

**Keywords:** wilms tumor, hub gene, risk stratification, prognostic model, nomogram

## Abstract

**Background:**

In children, Wilms’ tumors are the most common urological cancer with unsatisfactory prognosis, but few molecular prognostic markers have been discovered for it. With the rapid development of high-throughput quantitative proteomic and transcriptomic approaches, the molecular mechanisms of various cancers have been comprehensively explored. This study aimed to uncover the molecular mechanisms underlying Wilms tumor and build predictive models by use of microarray and RNA-seq data.

**Methods:**

Gene expression datasets were downloaded from Therapeutically Applicable Research to Generate Effective Treatments (TARGET) and Gene Expression Omnibus (GEO) databases. Bioinformatics methods wereutilized to identified hub genes, and these hub genes were validated by experiment. Nomogram predicting OS was developed using genetic risk score model and clinicopathological variables.

**Results:**

CDC20, BUB1 and CCNB2 were highly expressed in tumor tissues and able to affect cell proliferation and the cell cycle of SK-NEP-1 cells. This may reveal molecular biology features and a new therapeutic target of Wilms tumour.7 genes were selected as prognostic genes after univariate, Lasso, and multivariate Cox regression analyses and had good accuracy, a prognostic nomogram combined gene model with clinical factors was completed with high accuracy.

**Conclusions:**

The current study discovered CDC20,BUB1 and CCNB2 as hub-genes associated with Wilms tumor, providing references to understand the pathogenesis and be considered a novel candidate to target therapy and construct novel nomogram, incorporating both clinical risk factors and gene model, could be appropriately applied in preoperative individualized prediction of malignancy in patients with Wilms tumor.

## Introduction

Malignant renal tumors comprise 5% of all cancers occurring before the age of 15 years (1). The most common form of urologic cancer in children is Wilms tumor (2).Current treatment strategies *for* Wilms tumor include surgery, chemotherapy and radiotherapy. In high-income countries, 90% of patients with this tumor survive (3). While the OS in high, 20% of patients relapse after first-line therapy and up to 25% of survivors report severe late morbidity of treatment (4, 5).And the treatment of children with bilateral, high-risk tumors remains challenging (6). Novel biomarkers, therefore, are urgently needed in order to predict patients’ prognosis and develop novel target-specific therapies. But the introduction of biology-driven approaches to risk stratification and new drug development has been slower in Wilms tumor than in other childhood tumors (7).It is very important to improving prognosis for Wilms tumor patients by improving treatment based on clinical and biological risk factors, and further stratification of current treatment options based on tumor biology (6, 8).

The article "Identification of hub genes and construction of prognostic nomogram for patients with Wilms tumors" was retracted in 2023. Reasons: errors in the cell lines or tissues; unreliable results or conclusions; concerns about the data.

Many researchers are devoted to study about Wilms tumor. In the earlier study, Predisposition loci at 11p13(WT1),17q21(FWT1), 19q13 (FWT2) and 11p15 were identified by genetic linkage studies of familial Wilms tumor (9–11).With the development of modern genetic technology, the diverse genetic landscape of Wilms tumor is now beginning to be unveiled. Several of the variant genes that have been identified in Wilms tumor which are involved in histone modification during nephrogenesis (BCOR, MAP3K4, BRD7, CREBBP and HDAC4) (12). Recently, Putative predisposition genes include REST, CHEK2, EP300, PALB2 and ARID1A were identified (13, 14). Somatic mutations in SMARCA4, ARID1A, BCORL1, MAP3K4, NONO and MAX has also been discovered in Wilms tumor (15, 16). At present, there are several hot research topics like simultaneous allele loss of 1p and 16q, MYCN gain, loss of p53 function (17–20).These investigations provide novel insights to molecular mechanism of tumorigenesis and development of Wilms tumor. But the biological mechanism and prognostic effect still need further explore.

With the rapid advances in genomic and bioinformatics analysis, a large volume of cancer genomics data is being produced, benefiting cancer research. TARGET (Therapeutically Applicable Research to Generate Effective Treatments) aims to identify driver mutations and therapeutic targets for high-risk pediatric tumors through comprehensive integrative genomics (21). GEO (Gene Expression Omnibus) is another authoritative oncology database. Both of them comprised of massive sequencing data and clinic data about various tumors. Also, bioinformatics analysis of data matrix is widely used nowadays to determine differentially expressed genes (DEGs) and perform various analyses. By combining multiple databases, it is possible to integrate data from independent studies and obtain a greater number of samples for analysis, thus improving the rigor and accuracy of the results. Given the above, we integrated the patient data affected by Wilms tumor from TARGET and GEO database for further analysis by bioinformatics and experiments.

The article "Identification of hub genes and construction of prognostic nomogram for patients with Wilms tumors" was retracted in 2023. Reasons: errors in the cell lines or tissues; unreliable results or conclusions; concerns about the data.

In this study, we tried to identify hub genes to provide further insights into the occurrence and development of Wilms tumor. Also, we wanted establish a simple and effective model to predict the clinical classification and risk stratification of patients with Wilms tumor.

## Materials and methods

### Patients tissues and cell cultures

The RNA sequencing data and relating clinical information of Wilms tumor patients were downloaded from TARGET data portal (https://ocg.cancer.gov/programs/target). The inclusion criteria were as follows: (i) gene expression data of WT were available in the database; (ii) clinical data including gender, age, stage, and overall survival were complete; Finally, 125 patients were enrolled. For finding the Wilms tumor gene expression datasets,we performed systematic searches within the GEO database (https://www.ncbi.nlm.nih.gov/geo/). Three independent datasets were downloaded from GEO for further comprehensive analysis in this study, including GSE19249, GSE66405 and GSE73209 datasets. The GSE19249 include 6 tumor samples and 6 normal samples; the GSE66405 include 28 tumor samples and 4 normal samples; the GSE73209 include 32 tumor samples and 6 normal samples (**Table 1**).

**Table 1:** Details for 3 GEO dataset.

GSE	Authour	Platform	Tumour samples	Normal sample
**GSE19249**	Abdueva	[HG-U133_Plus_2] Affymetrix Human Genome U133 Plus	6	6
**GSE66405**	Ludwig	Agilent-039494 SurePrint G3 Human GE v2 8x60K Microarray 039381	28	4
**GSE73209**	Karlsson	Illumina HumanHT-12 V4.0 expression beadchip	32	6

This study comprised 13 patients with Wilms tumor who were diagnosed between 2011 and 2015. Tissue specimens were obtained from the pathology archives of the Sun Yat-Sen Memorial Hospital. Inclusion criteria were as follows: (1) lesions showing histologic features of Wilms tumor; (2) patients aged ≤14 years at the time of diagnosis; (3) availability of sufficient tissue for genomic assays; The study material included 18 formalin-fixed paraffin-embedded (FFPE) tissue specimens: primary tumors (n = 13), and normal tissues (n = 5).

SK-NEP-1 cell line were cultured in Dulbecco’s Modified Eagle’s medium (DMEM) supplemented with 10% fetal bovine serum (Bioind), streptomycin (100 μg/mL), and penicillin (100 μg/mL) (Gibco) and incubated at 37°C in a humidified chamber with 5% CO2.

The article "Identification of hub genes and construction of prognostic nomogram for patients with Wilms tumors" was retracted in 2023. Reasons: errors in the cell lines or tissues; unreliable results or conclusions; concerns about the data.

### Data pre-processing

Three series matrix files from GEO database were annotated with an official gene symbol using the data table of the microarray platform, and the gene expression matrix files were obtained respectively. The three gene expression matrix files were merged into one by Perl. Gene probes without gene symbols were eliminated and genes with more than one probe were averaged. To ensure the integrity and comparability of the datasets, the batch normalization of merged data was pre-processed by sva package using the R language (22). Patients’ mRNA expression data were downloaded from TARGET database and merged as one matrix through Perl software.

### Identification of DEGs and enrichment analysis

A package called Limma (3.18.2) from R Bioconductor was used to identify DEGs in GEO data matrix and TARGET data matrix respectively (23).The threshold of DEGs in the data set was set as the adjusted value of *p* < 0.05 and | log_2_FC| > 1 (FC: fold change). The FunRich software was used for analysis of DEGs that overlapped between the two databases and created the Venn diagram (24).Overlapping DEGs visualization was done using a volcano map and heatmap using gglot2 and the pheatmap package (25). We conducted gene ontology analysis (GO) and Kyoto encyclopedia of genes and genomes analysis (KEGG) using the ClusterProfiler package to further understand the overlapping DEGs potential biological processes, cell components, molecular function, and enrichment signaling pathways (26–28). It was deemed significant when p values were less than 0.05.

### Construction of protein-protein interaction network

The STRING website (http://string-db.org)was used to identify protein–protein interactions (PPIs) of the overlapping DEGs (29). The interactions with reliability scores more than 0.7 were selected for analysis. After that, Cytoscape software was used for PPI network analysis and visualization (30). we utilized the plugin MCODE to screen hub modules and cytoHubba to calculate the degree of genes in the PPI network and obtain the top 10 hub genes with the highest degree for further studies (31).

### qRT-PCR assay

Total RNA from 4 tumor tissues and 4 normal tissues was extracted by using TRIzol reagent. The specific steps were in strict accordance with the protocol. The Nanodrop 2000 UV spectrophotometer was used to detect the extracted RNA concentration and purity. Calculate the volume required for 100ng of RNA which were used for reverse transcription. The cDNA was synthesized by *reverse transcription* for further *experiments*. Primer sequences were designed and produced by Servicebio Company, The GAPDH gene was used as the reference control. *Reverse transcription* was performed in a total of 20ul volume containing 100 ng RNA, 3 *µl* 5x gDNA digester Mix, 5ul 4x HifairIII Supermix plus and RNase-free water supplemented to 20 µl. The reaction conditions were as follows: *25*°C for 5 min, 55°C for 15 min, 85°C for 5 min., 4°C ∞. The synthesized cDNA was stored *in* an ultra-low temperature *freezer* (−20°C). A total of 10 µl of the real-time PCR system was prepared containing: 2 µl of cDNA,1 µl of primer mix,5 µl of SYBR Green Master(Low Rox), and 2 µl of DEPC H_2_O supplemented. Cycling mode was set as: 40 cycles of 95 °C 15 s, 60 °C 30 s. Relative expression was analyzed using 2^−ΔΔCt^ method and GAPDH served as internal control. All experiments were conveyed in triplicates. Primer sequences are shown in **Table 2**.

The article "Identification of hub genes and construction of prognostic nomogram for patients with Wilms tumors" was retracted in 2023. Reasons: errors in the cell lines or tissues; unreliable results or conclusions; concerns about the data.

**Table 2:** Primers used for qRT-PCR.

Name	Sequence (5’-3’)
BUB1-F	TCATTCATGGAGACATTAAAC
BUB1-R	CTGAGCATCTCAACACACTG
CDC20-F	GCTTTGAACCTGAACGGTTTTG
CDC20-R	TCTGGCGCATTTTGTGGTTTT
CCNB2-F	CCGACGGTGTCCAGTGATTT
CCNB2-R	TGTTGTTTTGGTGGGTTGAACT
MAD2L1-F	GTTCTTCTCATTCGGCATCAACA
MAD2L1-R	GAGTCCGTATTTCTGCACTCG
KIF11-F	TATTGAATGGGCGCTAGCTT
KIF11-R	TCGTCTGCGAAGAAGAAAGA
PBK-F	AGACCCTAAAGATCGTCCTTCTG
PBK-R	GTGTTTTAAGTCAGCATGAGCAG
TOP2A-F	CTAGTTAATGCTGCGGACAACA
TOP2A-R	CATTTCGACCACCTGTCACTT
ASPM-F	GGCCCTAGACAACCCTAACGA
ASPM-R	AGCTTGGTGTTTCAGAACATCA
KIF2C-F	GTGTCTGTGTTAGGAAACGCCC
KIF2C-R	CACTTGCTAGGAATGGAAATCACAT
CDCA8-F	GAAGGGCAGTAGTCGGGTG
CDCA8-R	TCACGGTCGAAGTCTTTCAGA
H-GAPDH-S	GGAAGCTTGTCATCAATGGAAATC
H-GAPDH-A	TGATGACCCTTTTGGCTCCC

### IHC staining

A total of 20 formalin-fixed, paraffin-embedded biopsy tissues were available included 15 wilms tumor tissue and 5 normal tissues. The paraffin sections were deparaffinized by dimethylbenzene and rehydrated by graded alcohol. Then, *EDTA* antigen restore solution was used to repair antigens on slices in a microwave oven at the condition of moderate heat for 8 min, heat preservation for 8 min, and moderate-low heat for 8 min followed by natural cooling. After cooling, the sections were put in 0.3% hydrogen peroxide solution for 20 min to block endogenous peroxidase. After washing with PBS, blocking was performed with 3% BSA for 30 min at room temperature. The blocking solution was discarded, and *the* primary *antibody* was added and incubated overnight at *4*°C in a wet box. *The concentrations* used for *the primary antibodies were* at 1:50 (anti-BUB1, Abcam, ab195268), 1:200 (anti-CDC20, Abcam, ab183479) and 1:100 (anti-CNNB2, Abcam, ab15622) dilutions respectively. Following washes with *PBS*, a corresponding secondary antibody (1: 200, Servicebio, GB23303) was added, incubated at room temperature for 1 h, and washed with PBS.DBA solution was added, color development was checked under the microscope and the solution was washed with distilled water after satisfactory color development. Hematoxylin counterstain, water wash and wash fully with water after differentiation till *return blue*; routine dehydration and transparence; neutral gum mounting. Brownish yellow staining detected by microscopy indicated positive expression.

The article "Identification of hub genes and construction of prognostic nomogram for patients with Wilms tumors" was retracted in 2023. Reasons: errors in the cell lines or tissues; unreliable results or conclusions; concerns about the data.

### Oligonucleotide transfection

Small interfering RNAs (siRNAs) were purchased from GenePharma (Shanghai, China) based on the following sequences: BUB1‐specific siRNA: 5′‐GGCCUGCAUUUCUAAGAAUTT‐3′ (sense), 5′‐AUUCUUAGAAAUGCAGGCCTT‐3′ (anti‐sense); CDC20‐specific siRNA: 5′‐GGAAGACCUGCCGUUACAUTT‐3′ (sense), 5′‐AUGUAACGGCAGGUCUUCCTT‐3′(anti‐sense);CCNB2‐specific siRNA:5′‐GCAGCACAUGGCCAAGAAUTT‐3′ (sense), 5′-AUUCUUGGCCAUGUGCUGCTT‐3′(anti‐sense);NC: 5′‐UUCUCCGAACGUGUCACGUTT‐3′ (sense), 5′‐ACGUGACACGUUCGGAGAATT‐3′ (anti‐sense).Cell transfection was conducted using the Lipofectamine RNAiMax Transfection Reagent (Life Technologies).

### Cell proliferation assay

SK-NEP-1 cells were reseeded into 96-well plates (5 × 103 cells per well), and cell proliferation was assessed by the CCK-8 assay (Beyotime). The absorbance of each well was measured at a wavelength of 450 nm using a SPARK 10 M spectrophotometer (Tecan, Austria).

### 5-Ethynyl -2′ -deoxyuridine assays

EdU assays were performed with the Cell-Light EdU DNA Cell Proliferation Kit (RiboBio, Guangzhou, China). The cells (5 × 103 per well) were seeded into each well of a 96-well plate and incubated for 48 h. Next, the cells were incubated with 100 ul of EdU for 2 h, fixed with 500 μl of 4% paraformaldehyde, and stained with Apollo Dye Solution. DAPI staining was used to identify the nucleic acid. Images of the cells were obtained with an inverted fluorescence microscope (Carl Zeiss, Jena, Germany), and the proportion of EdU-positive cells was calculated.

### Cell cycle

For cell cycle assays, cells were fixed overnight at 4°C in 70% ethanol, stained with propidium iodide, and analyzed with a FACS can flow cytometer (BD Biosciences, San Jose, CA, USA) and ModFit 3.0 software (Verity Software House, Topsham, ME, USA).

### Construction of 7-gene prognostic model and nomogram

OS related DEGs were identified by univariate COX regression, *lasso* regression and multivariate *Cox* regression (P<0.05) (32, 33). Only genes with nonzero coefficients in the lasso regression model were chosen to further calculate the risk score. Using the formula below, we calculated the risk score for each patient: risk score = expression level of gene1 × j1 + expression level of gene2 × j2 + … + expression level of gene x × j x, where j represents the coefficient. As a cut-off value, the median risk score was used to subdivide Wilms tumor patients into two risk groups - a high-risk group and a low-risk group.

The article "Identification of hub genes and construction of prognostic nomogram for patients with Wilms tumors" was retracted in 2023. Reasons: errors in the cell lines or tissues; unreliable results or conclusions; concerns about the data.

Thereafter, the R package “survival” was used for Kaplan-Meier (KM) analysis to compare OS between the two groups. The R package “time ROC” was used for ROC curve analysis to evaluate the prognostic model’s specificity and sensitivity. In the AUC, 0.5 indicated no discriminating ability, while 1 indicated perfect discrimination. 7-gene prognostic model was constructed.

### Building a predictive nomogram

Univariate and multivariate Cox regression analyses were performed to identify the independent prognostic factors among 7-gene prognostic model and clinical characteristics to build the nomogram. ”rms” R package was used to assess the prognostic nomogram probability of 0.5-, 1-, and 3-year OS for TARGET-WT patients. The discrimination performance of the nomogram was quantitatively assessed by the C-index and the AUC

## Result and discussion

### Identification of overlapping DEGs

After data matrix from TARGET and GEO database were merged respectively, DEGs between normal and tumor were identified using R language. In total, 841 DEGs (635 downregulated and 206 upregulated mRNAs),5584 DEGs (4437 downregulated and 5327 upregulated mRNAs) were screened from the GEO data matrix and TARGET data matrix(**Figures 1A, B**). Among them, 688 DEGs overlapped; 191 were up-regulated, and 497 were down-regulated just like the Venn diagram show. Meanwhile, these overlapping DEGs were visualized in volcano plots (**Figure 1C**).

**Figure 1:** **(A)** and **(B)** Volcano plot of differentially expressed genes of Wilms tumor patients from GEO and TARGET database. Genes with P < 0.05 and logFC >1 or <-1 were considered as DEGs in each series. Blue, down-regulated genes; Gray, non-differential genes; Red, up-regulated genes **(C)** Venn diagram showing the intersection of the DEGs identified in two databases.

### Enrichment analysis of the overlapping DEGs

To explore the underlying biological process correlated to WT, the overlapping DEGs analysis were conducted using GO and KEGG enrichment analysis. For GO-biological process (GO-BP) enrichment analysis, the results showed that the genes involved in small molecule catabolic process, urogenital system development, renal system development etc. were significantly enriched. For GO-cellular component (GO-CC) enrichment analysis, the genes involved in apical part of cell, apical plasma membrane, basal plasma membrane, etc. were significantly enriched. For GO-molecular function (GO-MF) enrichment analysis, the genes involved in active transmembrane transporter activity, metal ion transmembrane transporter activity etc. were significantly enriched (**Figures 2A, B**). The results of the KEGG pathway analysis showed that the genes involved in Carbon metabolism, PPAR signaling pathway, etc. were significantly enriched (**Figures 2C, D**).

The article "Identification of hub genes and construction of prognostic nomogram for patients with Wilms tumors" was retracted in 2023. Reasons: errors in the cell lines or tissues; unreliable results or conclusions; concerns about the data.

**Figure 2:** Bar charts and bubble map of GO and KEGG pathway analyses. **(A)** GO enrichment bar chart of DEGs: The 10 most significant enriched terms in biological process, cellular component, and molecular function are select. **(B)** GO enrichment bubble map of DEGs. Bubble size represents the number of enriched genes, and bubble color difference represents the significance of target gene enrichment. **(C)** KEGG enrichment analysis bar chart of DEGs. The top 24 pathways from the KEGG enrichment analysis ranked by p-value. **(D)** KEGG enrichment bubble map of DEG.

### A total of 10 hub genes were selected by the PPI network

The STRING database was applied to construct a PPI network of these 688 genes to explore the core modules and hub genes that played the most importance in modular genes (**Figure 3A**). PPI network visualization was performed using Cytoscape. The plug-in MCODE in Cytoscape was used to detect the dense connection region of the molecular interaction network, of which had a high possibility of being involved in some important biological processes. Finally, a total of sixteen important modules were obtained, and the module with the highest score was screened out(**Figure 3C**); top 30 hub genes were screened out according to the node degree (**Figure 3B**).

**Figure 3:** Protein-protein interaction (PPI) network, hub gene screening, and hub cluster. **(A)** PPI network (688 DEGs filtered into the PPI network that contained 685 nodes and 1703 edges). **(B)** The predicted association rank (from low to high) of the top 30 genes in the PPI network. **(C)** The key modules identified using the MCODE plugin of Cytoscape, which contains 41 nodes/791 edges.

### Hub genes expression levels in Wilms tumor tissue and normal tissue

The expression of 10 hub genes in tumor and normal tissues was examined using Real-time PCR. Experiment was repeated more than *3* times. In tumor tissues compared with the normal tissues, the mRNA expression of CDC20 (<0.000001) 、CNNB2 (<0.01) 、BUB1(<0.0009) was significantly increased (**Figure 4A**). Statistical significance among samples was evaluated by paired t-test (*P<0.05).

**Figure 4:** CDC20, CCNB2 and BUB1 are highly expressed in tumor tissue. **(A)** Expression levels of CDC20, CNNB2 and BUB1 mRNA determined by real-time PCR in Wilms tumor (T) and normal (N) tissues. **(B)** Expression levels of CDC20,CNNB2 and BUB1 protein determined by IHC in Wilms tumor (T) and normal (N) tissues.

The article "Identification of hub genes and construction of prognostic nomogram for patients with Wilms tumors" was retracted in 2023. Reasons: errors in the cell lines or tissues; unreliable results or conclusions; concerns about the data.

Moreover, the protein level of CDC20、CNNB2、BUB1 was evaluated by IHC. Brown represents DAB positive immunoreactivity and the blue color is the hematoxylin counterstain. Results from immunohistochemistry showed that CDC20、CNNB2、BUB1 protein was upregulated in tumor tissue (**Figure 4B**).

### Effect of CDC20, CNNB2, and BUB1 knockdown on the proliferation of SK-NEP-1 cells

To determine the effect of CDC20, CNNB2, and BUB1 on SK-NEP-1 cells, CCK-8 and EdU assay was conducted in SK-NEP-1 cells following infection with si-CDC20, si-CNNB2, si-BUB1 and si-NC. The results revealed that CDC20 and CNNB2 knockdown significantly inhibited the proliferation of Wilms tumor cells (*** *p* < 0.001, ** *p* < 0.01, * P<0.05; **Figures 5A-D**).

**Figure 5:** CDC20, CNNB2, and BUB1 affects the proliferation of SK-NEP-1 cells. **(A-D)** The cell proliferative ability was assessed by the Cell Counting Kit-8 (CCK-8), and EdU assay after CDC20, CNNB2, and BUB1 was knocked down in SK-NEP-1 cells. **(E-H)** Down-regulation of CDC20, CNNB2, and BUB1 arrests the cell cycle of SK-NEP-1 cells(**P < 0.01, ns, none sense).

### Effect of CDC20, CNNB2, and BUB1 knockdown on the cell cycle of Wilms tumor cells

To further investigate the role for CDC20, CNNB2, BUB1in tumor growth, a cell cycle analysis was performed using flow cytometry. SK-NEP-1 cells infected with si-CDC20, si-CNNB2, si-BUB1 and si-NC exhibited a notable increase in the percentage of cells in the G0/G1 phase compared with the si-NC groups. the proportion of cells in the S phase showed a variable change depending on the cell type, and the proportion of cells in the G2/M phase also significantly decreased (**Figures 5E-H**).

### Establishment of the 7-gene-based prognostic model in Wilms tumor patients

Univariate *Cox* regression was performed and a total of 43 *OS*-related genes were identified. To construct a more practical model, we employed LASSO regression to screen the most reliable predictive prognostic genes from the above 43 genes, including FCN3, CDC20, and E2F1. The optimal gene model consisting of 18 prognosis DEGs, at the same time, the corresponding coefficients were identified (**Figure 6A**). Multivariate *Cox* regression analysis further screened 7 prognosis-related genes out of the 18 prognosis-related genes identified from *Lasso* regression analysis. Of the 7 genes identified, HPD and PRC1 were found to be associated with a high risk, showing a HR of >1, whereas CYP27C1,HEY1,EGF,ASPA and TMEM61 were identified as a low-risk gene, with HR <1.

The article "Identification of hub genes and construction of prognostic nomogram for patients with Wilms tumors" was retracted in 2023. Reasons: errors in the cell lines or tissues; unreliable results or conclusions; concerns about the data.

**Figure 6:** Construction of gene prognostic models and their prognostic characteristics. **(A)** Eighteen genes were used to construct the risk models. Coefficients were calculated from univariate Cox regression analysis using LASSO. **(B)** Survival analysis was performed using the Kaplan‐Meier method for the overall survival of patients in TARGET. **(C)** The predictive efficiency of the gene prognostic model showed by ROC curves based on 1-, 3‐ and 5‐year survival rates.

In order to validate the predictive capability of prognostic model, survival curves were generated by K*-*M survival analysis. Result showed that the predicted survival time of the high-risk group was significantly shorter (P<0.05) (**Figure 6B**). The 1-,3- and *5*-year survival rates of the high-risk group were 83.8%(95%CI=75%-93.5%),42.7%(95%CI=31.7%-57.5%)and 38.8%(95%CI=28%-58.8%), respectively, whereas those of the low-risk group were 93.6%(95%CI=87.8%-99.9%),86.9%(95%CI=78.9%-95.8%)and 81.3%(95%CI=71.9%-92%), respectively. The prediction capability of the risk score model was evaluated by calculating the area under the *ROC* curve. The 1*-, *3-, and 5-years AUC values were 0.727,0.820 and 0.817, respectively (**Figure 6C**).

### Establishment of nomogram

As shown in **Table 3**, univariate and multivariate Cox regression analyses showed that the ender, clinical stage and gene risk score were independent prognostic factors for OS. A nomogram was plotted based on those factors. The C-index was 0.766. The AUC values of the nomogram for predicting 1-,3- and 5-year OS were 0.828,0.837 and 0.827, respectively (**Figure 7A, B**). To further test the predictive power of the nomogram, ROC curves were drawn to compare the predictive performance between the nomogram and the other 3 independent predictors. The nomogram obtained the highest 1-,3- and 5- year area under the curve (**Figures 8A–C**).

**Table 3:** Univariate and multivariate Cox regression analysis of different prognostic variables for overall survival (OS) prediction in Wilms tumor patients.

Characteristic	Univariate Cox regression		Multivariate Cox regression	
	HR (95%CI)	P value	HR (95%CI)	P value
Age (years)		0		0
0-3	1		——	——
3-6	1.6326 (0.8349, 3.193)	0.152	——	——
>=6	0.7386 (0.3018, 1.808)	0.507	——	——
Gender		0		0
Female	1		1	
Male	1.785 (1.023, 3.114)	0.0414	2.138 (1.205, 3.793)	0.00936
Clinic stage		0		0
I-II	1		1	
III-IV	3.059 (1.686, 5.551)	0.000235	3.513 (1.898, 6.499)	6.28E-05
Gene risk score		0		0
Low risk	1		1	
High risk	4.616 (2.44, 8.731)	2.56E-06	4.438 (2.330, 8.454)	5.81E-06

**Figure 7:** Nomogram and its AUC. **(A)** A prognostic nomogram predicting 1-, 2-, and 3-year overall survival of Wilms tumor patient. **(B)** ROC curve for 1-, 3-, and 5-year overall survival predictions for the nomogram.

The article "Identification of hub genes and construction of prognostic nomogram for patients with Wilms tumors" was retracted in 2023. Reasons: errors in the cell lines or tissues; unreliable results or conclusions; concerns about the data.

**Figure 8:** The AUC was used to estimate the predictive power of different models. (**A** ROC for 1 year; **B** ROC for 3 years; **C** ROC for 5 years). The predictive ability of the nomogram (purple,1-,3-,5- year AUC= 0.828,0.837,0.827) was better than those of the other risk models.

## Discussion

Wilms tumor (*nephroblastoma*) *is* one of *the most common* pediatric solid tumors, and the survival rate of high*-*risk patients and relapsed patients is low. It is an urgent need to refine risk stratification and find a reliable biomarker for Wilms tumor patients.

In this study, the results of bioinformatics analysis predicted that BUB1, CCNB2 and CDC20 are hub genes of Wilms tumor, and this prediction was further proved by the experimental validation. The results proved that CDC20, CNNB2, and BUB1 was upregulated in Wilms tumor and significantly associated with the survival of Wilms tumor patients. Downregulation of CDC20 and CNNB2 markedly suppresses cell growth in cultured SK-NEP-1 cells which was consistent with the results of the functional prediction above. We determined with the cell cycle distribution analysis that the lack of CDC20, CNNB2, and BUB1 led to a G0/G1 phase arrest. We also tried to investigate how CDC20, CNNB2, and BUB1 participates in the development of Wilms tumor.

CDC20 is a cell cycle regulating protein (34). Various malignancies were reported overexpression of CDC20 and high expression of CDC20 was associated with higher tumor grade in bladder, cervical, colon, endometrial, gastric, liver, ovarian, prostatic, and renal carcinomas (35). In cells, BUB1 plays a crucial role in chromosome assembly and kinetochore localization (36).Bub1 also is a specific kinase optimized for CDC20 phosphoryation. CDC20 is the only known physiologically relevant substrate of BuB1 (37). CCNB2 is key protein of the cyclin family and regulates the progression of the G2/M transition during the cell cycle (38). According to Shubbar et al, breast cancer patients’ prognoses are affected by CNNB2 overexpression (39). Follow-up analysis has shown that CNNB2 overexpression is associated with poor prognosis. Li et al. found that CCNB2 overexpression in HCC is associated with poor prognosis, and knock-down of CCNB2 inhibits cell proliferation and migration, promotes apoptosis, and causes S phase arrest in HCC cell lines (40). Therefore, more comprehensive studies about molecular mechanism will remain to be lucubrated in the future.

Furthermore, to identify potential gene biomarkers we investigated the differences in gene expression between tumor and normal tissues from Wilms tumor. The differentially expressed genes were screened, and univariate, Lasso and multivariate Cox analyses were used to build a risk model to predict Wilms tumor prognosis. We identified seven genes: PRC1, CYP27C1, HEY1, EGF, HPD, ASPA and TMEM61. Poor prognosis was associated with high levels of PRC1,CYP27C1 and HEY1 expression in Wilms tumor patients. In S. pombe, PCR participates in meiotic recombination, maintenance of heterochromatin structure, and regulation of certain genes related to sexual differentiation, besides induction of stress-responsive genes under oxidative, heat, reductive, osmotic, and starvation stresses with ATF1 by forming a heterodimer (41, 42) There are few studies on the CYP27C1 gene. CYP27C1 was a member of the cytochrome P450 superfamily of enzymes, which can catalyze a number of reactions associated with drug metabolism (43, 44). Some studies have indicated that CYP27C1 can convert vitamin A1 into A2, The CYP27C1-mediated vitamin A1-to-A2 switch could be a switch for visual sensitivity (44). In Bhavsar-Jog, CHRM1, CYP27C1 and FOXH1 are all linked to pathways related to Alzheimer’s disease (45). A deeper understanding of CYP27C1 is needed. HEY1 It was found that the AUCs of the ROC curves for the prognostic model to predict the 1,3 and 5‐year survival were0.727,0.820 and 0.817, respectively, indicating that the 7-gene signature performed well for survival prediction.

The article "Identification of hub genes and construction of prognostic nomogram for patients with Wilms tumors" was retracted in 2023. Reasons: errors in the cell lines or tissues; unreliable results or conclusions; concerns about the data.

The nomogram is a widely used prognostic evaluation tool in clinical oncology that can incorporate a variety of prognostic determinants, including molecular and clinicopathological findings (46). In our study, by combining gene signatures and clinic variables, a nomogram is developed to predict OS and to assist clinicians in making personalized treatment decisions. The predictive performance of the nomogram built with the combined model is the best by C‐index, AUC and compared with other single risk factor. The best performance of nomogram was confirmed.

The current study has several limitations that should be considered. First, the main information on clinical characteristics and gene expression data for the most part came from white, black or Hispanic populations; so the extrapolation of the findings to other ethnic groups needs to be established. Second, the nomogram was only performed using the TARGET database due to the lack of complete clinical information in other datasets; hence, the nomogram should be further validated through multicenter clinical trials and prospective studies. Third, the molecular mechanisms of the genes identified here and their roles in the pathogenesis and progression of Wilms tumor require further experimental studies. Certainly, future research will have to be done on refining these limitations.

The article "Identification of hub genes and construction of prognostic nomogram for patients with Wilms tumors" was retracted in 2023. Reasons: errors in the cell lines or tissues; unreliable results or conclusions; concerns about the data.

## Conclusion

Our study discovers three critical gene signatures of Wilms tumor, they are CDC20, BUB1 and NNB2. They could serve as the basis for subsequent experimental analysis. The prognostic models constructed by nomogram produce more effective predictions.

## Data availability statement

The datasets presented in this study can be found in online repositories. The names of the repository/repositories and accession number(s) can be found in the article/supplementary material.

## Ethics statement

The studies involving human participants were reviewed and approved by Sun Yat-Sen Memorial Hospital. Written informed consent to participate in this study was provided by the participants’ legal guardian/next of kin. Written informed consent was obtained from the individual(s), and minor(s)’ legal guardian/next of kin, for the publication of any potentially identifiable images or data included in this article.

## Author contributions

XD and LL conceived and designed the study. LL performed bioinformatic analysis; LC and LL performed the experiments. DG, LL and LC wrote and critically reviewed the manuscript. All authors discussed the results and commented on the manuscript. All authors read and approved the final manuscript.

## Funding

This work was supported by Guangzhou Production, Education and Research collaborative innovation major project (Projects of people’s livelihood) (No.201604020151),the Natural Science Foundation of Guangdong Province (No.2015A030313037, No.2022A1515012222) the Municipal School Joint Project of Guangzhou Science and Technology Bureau (104287750039) Funding by Science and Technology Projects in Guangzhou(202201020395) and the Guangdong Provincial Science and Technology Plan Project (2014A020213021).

## Conflict of interest

The authors declare that the research was conducted in the absence of any commercial or financial relationships that could be construed as a potential conflict of interest.

## Publisher’s note

All claims expressed in this article are solely those of the authors and do not necessarily represent those of their affiliated organizations, or those of the publisher, the editors and the reviewers. Any product that may be evaluated in this article, or claim that may be made by its manufacturer, is not guaranteed or endorsed by the publisher.
